# miR-122 Regulates Tumorigenesis in Hepatocellular Carcinoma by Targeting AKT3

**DOI:** 10.1371/journal.pone.0079655

**Published:** 2013-11-07

**Authors:** Rounak Nassirpour, Pramod P. Mehta, Min-Jean Yin

**Affiliations:** Oncology Research, Pfizer Worldwide Research and Development, San Diego, California, United States of America; H.Lee Moffitt Cancer Center & Research Institute, United States of America

## Abstract

MicroRNAs (miRNAs) have been implicated in the orchestration of diverse cellular processes including differentiation, proliferation, and apoptosis and are believed to play pivotal roles as oncogenes and tumor suppressors. miR-122, a liver specific miRNA, is significantly down-regulated in most hepatocellular carcinomas (HCCs) but its role in tumorigenesis remains poorly understood. Here we identify AKT3 as a novel and direct target of miR-122. Restoration of miR-122 expression in HCC cell lines decreases AKT3 levels, inhibits cell migration and proliferation, and induces apoptosis. These anti-tumor phenotypes can be rescued by reconstitution of AKT3 expression indicating the essential role of AKT3 in miR-122 mediated HCC transformation. In vivo, restoration of miR-122 completely inhibited xenograft growth of HCC tumor in mice. Our data strongly suggest that miR-122 is a tumor suppressor that targets AKT3 to regulate tumorigenesis in HCCs and a potential therapeutic candidate for liver cancer.

## Introduction

MiRNAs are small non-coding RNAs that act as agents of the RNA interference pathway to regulate protein expression by destabilization and/or translational inhibition of target messenger RNAs (mRNAs) [1]. Because miRNAs usually bind to their targets with incomplete complementarity, one single miRNA may have multiple gene targets and numerous effectors within the same functional pathway, producing a coherent physiological response via multiple parallel perturbations [2], [3]. In fact, miRNAs have been implicated in the regulation of a variety of complex biological functions including cellular proliferation, differentiation and apoptosis and are therefore attractive cancer therapeutic targets [4], [5]. Additionally, miRNAs are frequently located at fragile sites and genomic regions susceptible to amplification, deletion, or translocation during tumor development [6] and growing evidence suggests that miRNAs can function as tumor suppressors or oncogenes [4]. Interestingly miRNA expression profiling analyses have revealed characteristic miRNA signatures for various human cancers [7], [8].

Hepatocellular carcinoma (HCC) is the fifth most common human cancer, affecting over 500,000 people each year worldwide with major risk factors such as hepatitis B and C infections, alcohol abuse, xenobiotics, primary billiary cirrhosis, diabetes, non-alcoholic fatty liver disease, and genetic disorders such as hemochromatosis and α1-antitrypsin deficiency [9]. Although recent advances in functional genomics provide an increasingly comprehensive understanding of hepatocarcinoma development [10], [11], the molecular pathogenesis of HCC remains poorly understood and the clinical heterogeneity of HCC combined with lack of sensitive and early diagnostic biomarkers and treatment strategies have led to a high mortality rate for HCC patients. Therefore, research and development for effective targeted therapies are in strong need to combat this aggressive cancer.

miR-122 is the most abundant miRNA in the liver, constituting 70% of the total hepatic miRNAs [12], [13]. Not only is miR-122 crucial to normal liver development and function, including fatty acid and cholesterol metabolism, but it also seems to play pivotal roles in various liver diseases such as the Hepatitis C Virus (HCV) replication [14], [15]. Additionally, this liver specific miRNA has been reported to be dramatically down regulated in most HCCs, where it is often inversely associated with poor prognosis and metastasis [16]–[18]. In fact, mice with germline knockout or liver specific knockout of miR-122 develop steatohepatitis, fibrosis and spontaneous tumors resembling HCC [19], [20]. Although Cyclin G1, MDR, ADAM17, and CUTL1 have been proposed as targets of miR-122, the mechanism behind miR-122 regulation of tumorigenesis in HCCs remains poorly understood [18], [21]–[23].

In this study, we identify AKT3 as a novel and direct target of miR-122 in human HCCs. In summary, our data demonstrate that AKT3 expression is inversely correlated to miR-122 levels in HCC cell lines, and that over-expression of miR-122 in a subset of HCC cell lines decreases AKT3 mRNA and protein levels by directly binding to the 3’UTR of AKT3, which subsequently leads to inhibition of cell proliferation and migration. Consequently, we were able to rescue these miR-122 induced anti-tumor activities by reconstituting AKT3 expression. *In vivo*, over-expression of miR-122 in a HCC cell line, SNU-182, also inhibited xenograft tumor growth in nude mice. Therefore, our data strongly suggest that miR-122 is a tumor suppressor by targeting AKT3 expression to modulate HCC cell transformation, and that over-expression of miR-122 or down-regulation of AKT3 may prove beneficial as therapeutic potentials for HCC patients.

## Results

### miR-122 directly binds to the 3’UTR of hs-AKT3 to regulate its expression

We first confirmed that miR-122 is exclusively expressed in normal human liver tissue by comparing its expression in other normal tissues (Figure 1A). miR-122 expression in tumor cell lines from other organs was very low (Figure 1B), further confirming that miR-122 is a liver-specific miRNA as reported. Using real-time RT-PCR, we also confirmed that miR-122 expression was significantly down-regulated or completely abolished in a variety of human HCC cell lines including Hep-3B2, SNU-182, SNU-475, as well as a hepatoblastoma cell line Hep-G2. Although the HCV-transformed HCC cell line Huh-7 also showed reduced expression of miR-122, it still maintained a significant level of miR-122 expression, as shown in Figure 1B. Therefore, miR-122 expression is specific to liver and is highly suppressed in the human HCC cell lines tested.

**Figure 1:** miR-122 is down regulated in human hepatocellular carcinoma cell lines. (**A**) miR-122 level, normalized to RNU-48, was measured in RNA samples collected from normal stomach, lung, colon, and breast tissues. (**B**) Normalized miR-122 expression in a variety of human cancer cell lines.

Next we searched bioinformatic prediction algorithms such as miRanda, TargetMiner, DIANA-MicroT, UPennrna22, and miRDB for predicted targets of this miRNA. AKT3 was identified as one of the candidate targets for hsa-*miR*-*122-5p*. Using a different bioinformatic algorithm, Tsai and colleagues also had previously listed AKT3 *a*s a potential target of miR*-*122, although they did not explore this interaction [18]. Since AKT is a key regulator in many cancers, we decided to investigate the sequence alignments between AKT3 3’UTR further, and found that in three species, the human miR-122 in fact shows partial complementarity (Figure 2A). We then amplified the human AKT3 3’UTR by PCR and sub-cloned it into a luciferase reporter vector as illustrated in Figure 2B. This construct was used for co-transfection with miR-122 construct in SNU182 (cells lacking endogenous miR-122 expression) and Huh7 (cells harboring some endogenous miR122 expression) cell lines. A luciferase assay was then used in determining whether miR-122 can bind to the 3’UTR of AKT3. Results demonstrate that miR-122 expression remarkably decreased the firefly luciferase activity in SNU-182 cells indicating miR-122 binding to 3’UTR (Figure 2C). As expected, we observed a lower basal firefly luciferase activity in Huh-7 relative to SNU-182, due to the endogenous expression of miR-122 in Huh-7 cells, as indicated in Figure 1B. Transfection of miR-122 into Huh-7 cells did however decrease the luciferase activity, albeit to a lower degree (Figure 2C). Since the 3’UTR of the other 2 members of the mammalian AKT family, AKT1 and AKT2, lack any predicted binding sites for miR-122, we focused our binding luciferase assays on the AKT3-isoform. Therefore, the luciferase reporter assay confirms direct binding of miR-122 to hsa-AKT3 3’UTR.

**Figure 2:** miR-122 directly binds to the 3’UTR of hsa-AKT3. (**A**) Sequence alignments of miR-122 with 3’UTR of AKT3 from 3 mammalian species shows partial complementarity. (**B**) Schematic representation describing the 3’UTR luciferase reporter assay. The assay was carried out simultaneously in SNU-182 and Huh-7 cells, over-expressing miR-122 GFP or the GFP vector alone, as well as parental cells co-transfected with the pGL3-3’UTR construct containing AKT3 3’UTR. Luciferase assays were performed 48 hours after transfection using the Dual-Luciferase Reporter Assay System (Promega). Firefly luciferase activity was normalized to Renilla luciferase activity to account for variations in transfection efficiency. Firefly luciferase activity will be reduced if there is a direct binding between miR-122 and the 3’UTR of AKT3 sequence inserted in the vector. (**C**) Luciferase activity was measured in SNU-182 and Huh-7 parental, miR-122-GFP and GFP over-expressing cells transfected with the luciferase reporter 3’UTR construct or vector alone. Results represent at least three different independent experiments, and statistical significance between indicated groups is depicted as ** *P*<0.01, *** *P*<0.005.

### AKT3 expression is inversely correlated to miR-122 levels in HBV transformed HCC cell lines

We next examined the expression levels of miR-122 and AKT3 in the normal human liver and human HCC cell lines. As shown in Figure 1 and Figure 3A, miR-122 expression is greatly reduced in the HCC cell lines compared to that in normal liver. Concurrently, AKT3 expression level is up-regulated in all three HCC cell lines (Hep3B2, SNU-182 and SNU-475) with little or no expression of miR-122 (Figure 3A). Interestingly, in the hepatoblastoma HepG2 cells and the HCV-transformed Huh-7 lines, AKT3 is not over-expressed in comparison to normal liver tissue (Figure 3A). The Huh-7 AKT3 levels are not surprising considering the endogenous expression of miR-122 in these cells. As expected due to a lack of miR-122 binding site, although highly homologous, AKT1 and AKT2 mRNA levels only showed slight increases in the HCC cell lines in comparison to normal liver (Figure 3B). Similar to the observations made for AKT3 transcript levels, AKT3 protein levels were also significantly higher in SNU-182 and SNU-475 HCC cell lines (Figure 3C). These results indicate that miR-122 level is inversely correlated to the AKT3 mRNA and protein levels in the HCC cell lines.

**Figure 3:** AKT3 expression is inversely correlated to miR-122 levels in HCC cell lines. (**A**) The AKT3 transcript level normalized to its expression in normal liver (right Y axis) and normalized miR-122 expression (left Y axis) were measured in various HCC cell lines. (**B**) The relative expression level of closely homologous isoforms AKT1 and AKT2 were measured in HCC cell lines. (**C**) Western blot analysis of total AKT and AKT3 protein levels in various HCC cell lines. Actin was used as the loading control in these studies.

### Over-expression of miR-122 in HCC down-regulates AKT3

We next examined the effects of miR-122 over expression in human HCC cell lines, SNU-182, SNU-475, Hep3B2, and Huh-7. miR-122 was sub-cloned in a lentiviral expression vector and was successfully over expressed in these cell lines (Figure 4A). As expected, over-expression of miR-122 decreased both the mRNA and protein levels of AKT3 in SNU-182 cells as shown in Figure 4A. Similar data was collected from the SNU-475, and Hep3B2 (data not shown). In Huh-7 cells, which express some endogenous miR-122, over-expression of miR122 also decreased AKT3 protein levels but this change was only visible on the immunoblot with long exposure time due to the low endogenous AKT3 levels in this cell line (Figure 4A). To confirm specificity, we also examined alterations in the other 2 AKT family members in these miR122 transduced cells. Over-expression of miR-122 in SNU-182 and Huh-7 did not significantly alter the AKT1 or AKT2 expression, as shown in Figure 4B, again suggesting that miR-122 specifically targets AKT3. Therefore, these results support the hypothesis that miR-122 negatively regulates AKT3 translation in HCC cell lines.

**Figure 4:** Restoring miR-122 expression decreased AKT3 translation. (**A**) AKT3 mRNA and protein levels were measured in SNU-182 and Huh-7 cells stably over-expressing miR-122-GFP or GFP alone. The membrane blot of the Huh-7 cells required unusually long exposures before the AKT3 bands could be visualized. (**B**) AKT1 and AKT2 transcript levels were measured in SNU-182 and Huh-7 cells stably over-expressing miR-122-GFP or GFP alone.

### Over-expression of miR-122 inhibits cell migration and induces apoptosis

AKT kinases regulate diverse cellular processes including cell proliferation and survival, cell size and response to nutrient availability, as well as tissue invasion and angiogenesis in both normal and tumor cells [24]. Since AKT3 is highly expressed in SNU-182 and SNU-475 cells (Figure 3), it is likely that AKT3 plays an essential role in the tumorigenesis of these cell lines. Therefore, we next investigated whether inhibition of AKT3 by restoring miR-122 expression would have anti-tumor effects in SNU-182 and SNU-475 in comparison to a HCC cell line (Huh-7) with endogenous miR122 expression. SNU-182, SNU-475, and Huh-7 cells are able to migrate across the polycarbonate membrane upon HGF-1 stimulation, a well established characteristic of highly transformed HCC cells. Over-expression of miR-122 decreased the HGF-induced cell migration in the HBV-transformed SNU-182 and SNU-475 but not in the HCV-transformed Huh-7 cells (Figure 5A) indicating the critical role of AKT3 in regulating migration in SUN-182 and SNU-475 cells. Since Huh7 already expresses miR-122, over-expression of this miRNA did not alter cell migration in these cells. To confirm that miR-122 induced inhibition in cell migration is due to the decreased level of AKT3 in SNU-182 and SNU-475 cells, we performed a rescue experiment by transiently transfecting a vector encoding the human AKT3 cDNA in the SNU-182 cells, which stably expressed GFP or miR-122-GFP. Results shown in Figure 5B clearly indicate that transient over expression of AKT3 in miR-122-GFP expressing SNU-182 cells rescues the migratory inhibition described above by approximately 70%. Taken together, the migration assays suggest that miR-122 over-expression in SNU-182 cells down regulates AKT3, which in turn inhibits the HGF-induced cell migration in these cells. Furthermore, these miR-122 inhibited migratory responses were rescued by partial restoration of AKT3 expression. Therefore, miR-122 regulation of AKT3 expression is necessary and sufficient in modulating HCC cellular migration in HBV-transformed cells.

**Figure 5:** Restoring miR-122 expression in HBV-transformed HCC cell lines inhibited cell migration and induced apoptosis. These miR122 induced anti-tumor activities were rescued by ectopic expression of AKT3. (**A**) Cell migration assays were performed on SNU-182 or Huh-7 cells over-expressing miR-122 GFP or GFP alone. Migratory responses to the bottom chamber with and without addition of stimulator (10% HGF) are shown. (**B**) Cell migration assays were performed using miR-122-GFP or GFP alone over-expressing SNU-182 cells with or without AKT3 reconstitution. (**C**) Phosphorylation of BAD, total BAD level and cleaved caspase 3 were measured in SNU-182 and Huh-7 cells over-expressing miR-122-GFP or GFP alone. (**D**) Transient reconstitution effects of AKT3 in SNU-182 cells over-expressing miR-122-GFP or GFP alone were also measured. Statistical significance between the indicated groups is depicted as *** *P*<0.005.

AKT family members have also been shown to regulate the apoptotic pathways mainly by a phosphorylation dependent inhibition of the pro-apoptotic Bcl-2 family member, BAD, to promote cell survival [25]. We had noticed that the HCC cells transduced with miR-122 showed slower growth rates in culture relative to their parental cell lines. Therefore, we next studied the effects of miR-122 over-expression on apoptosis/proliferation. SNU-182 cells over-expressing miR-122 exhibited decreased phosphorylation of BAD, in addition to an increase in total BAD levels in comparison to the parental cells and Huh-7 cells over-expressing miR-122 (Figure 5C). Furthermore, HBV-transformed cell lines SNU-182 and Hep-3B2 (data not shown) cells over-expressing miR-122 showed elevations of cleaved caspase 3 levels, another pro-apoptotic protein marker (Figure 5C). These data indicate that restoration of miR-122 in HCC cell lines mediates phosphorylation and up-regulation of BAD to promote apoptosis in SNU-182 cells but not in Huh-7 cells, which endogenously express miR-122. To further confirm that the decreased pBAD and increased cleaved caspase 3 in miR-122 over-expressing SNU-182 cells is due to AKT3 down regulation, AKT3 rescue experiments were performed and data showed that ectopic transient expression of AKT3 is able to partially rescue the effects of miR-122 over-expression in SNU-182 cells (Figure 5D). These data taken together strongly suggest that miR-122 over-expression in SNU-182 cells decreases cell migration and increases apoptosis through its direct regulation of AKT3 translation.

### Over-expression of miR-122 induces in-vitro as well as in-vivo anti-tumor activities in aggressive HCC cell line, SNU-182 cells

After establishing the modulation of the apoptotic pathways by miR-122 in HCC cell lines, we next explored the effects of miR-122 on cell proliferation. As expected and in agreement with our apoptotic assays, over expression of miR-122 dramatically slowed down cell proliferation in SNU-182 but not in Huh-7 cells (Figure 6A and 6C). The inhibition of cell proliferation was rescued by ectopic expression of AKT3 in miR-122 harboring SNU-182 cells (Figure 6B). The lack of regulation observed in Huh-7 cells with miR-122 over-expression could again be contributed to the maintained endogenous miR-122 expression in these cells indicating that increasing miR-122 expression in these cells is not sufficient to alter their tumorigenic abilities. We finally investigated the effects of miR-122 over-expression on *in-vivo* tumor growth. SNU-182 cells stably over-expressing miR-122-GFP were established and subcutaneously implanted in nude mice, and tumor growth was monitored over time (SNU182 cells stably expressing GFP alone as well parental cell lines were used as control). Figure 6D shows a dramatic reduction in tumor growth in miR-122 over-expressing SNU-182 xenograft models. Therefore, over-expression of miR-122 in the highly transformed SNU-182 HCC cell line induced *in-vitro* and *in-vivo* anti-tumor activity classifying miR-122 as a HCC tumor suppressor.

**Figure 6:** miR-122 over-expression inhibited *in-vitro* cell proliferation and *in-vivo* tumor growth in a highly transformed HCC SNU-182 xenograft mouse model. Cell proliferation was measured in (A) SNU-182 and (C) Huh-7 parental cells and cells stably over-expressing miR-122-GFP or GFP alone. (B) Cell proliferation was measured in SNU-182 cells over-expressing miR-122-GFP or GFP with or without the reconstitution of AKT3 expression. (D) Nude mice were implanted with SNU-182 parental lines as well as cells over-expressing miR-122-GFP or GFP vector alone, and tumor growth was monitored and plotted as tumor volume (mm^3^) over time. Statistical significance between the indicated groups are depicted as ** *P*<0.01, and *** *P*<0.005.

## Discussion

miR-122 has previously been shown to be dramatically down regulated in most HCCs and is generally indicative of poor prognosis and higher risk of metastasis [16]–[18]. This study investigates the role of miR-122 in the tumorigenesis of HCCs. Here we show that miR-122 functions as a tumor suppressor in the HBV-transformed HCC human cell lines and report AKT3 as a novel and direct target of miR-122. Importantly, restoring miR-122 expression suppresses HCC cell migration and in vivo tumor growth and induces apoptosis by its direct and specific regulation of AKT3.

Although several targets have been reported for miR-122 to date [18], [21]–[23], none can fully account for the wide range of cellular transformation and tumorigenic characteristics observed in the miR-122 down regulated HCCs. AKT, also known as Protein Kinase B (PKB), is a serine/threonine kinase that plays a key role in multiple cellular transformation processes such as apoptosis, cell proliferation, and cell migration. In this study, we demonstrate that miR-122 directly targets AKT3 to regulate the cellular transformations and tumorigenesis in non-HCV transformed human HCC cell lines (Figure 2). Furthermore, restoring miR-122 expression in these cell lines not only induced apoptosis and inhibited migration, but also dramatically suppressed tumorigenesis. Since the phenotypes induced by miR-122 over expression were rescued by a transient expression of ectopic AKT3, we propose that miR-122 regulation of AKT3 expression is necessary and sufficient for modulating tumorigenesis and cellular transformation in human HCC cell lines.

The AKT family is comprised of three closely related isoforms: AKT1, AKT2, and AKT3, which have a highly conserved domain structure and presumably play similar roles in cell proliferation, survival, metabolism, and many other cellular functions [26]. However, there are functional distinctions among the AKT isoforms in mediating tumor development and progression which seems to be orchestrated in a tissue specific manner [27], [28]. Gene knockout and siRNA studies on AKT1 and AKT2 have revealed isoform-specific functions of AKT family members in their regulation of cell migration, which generally correlate with tumor invasiveness and metastasis. Interestingly, very little is known regarding the role of AKT3 in cell migration [27]. Additionally, although all three AKT isoforms are able to transform cells *in-vitro* [29], amplification or gene mutation of AKT3 have not been reported in human cancers [26]. A growing number of recent publications suggest that HBV enhances the expression of the mTOR and PI3K/Akt pathways (e.g. Wang et al. 2013). In this study, we show that the HBV transformed cells show both significantly decreased miR-122 expression as well as an enhanced expression of AKT3 which seems to regulate tumorigenesis in this subclass of highly aggressive and transformed HCCs. Our data clearly demonstrate that targeting and specific down-regulation of AKT3 by miR-122 over expression (as shown in Figure 4B) was able to block migration and this inhibition was rescued by reconstitution of AKT3 expression. Interestingly, sustained AKT1 and AKT2 expression in SNU-182 cells was not sufficient in maintaining cell migration in miR-122 over-expressing cells, suggesting that AKT3, but not AKT1 or AKT2, is necessary and sufficient in regulating migration and metastasis in some HCCs.

AKT family members are also established regulators of apoptosis. They can promote growth factor-mediated cell survival both directly and indirectly by phosphorylating a variety of apoptotic substrates, such as Bad, a pro-apoptotic Bcl-2 family member [25]. AKTs have been shown to phosphorylate Bad, which in turn inhibits its pro-apoptotic functions to promote cellular proliferation and decreases caspase activity. Not surprisingly, down regulation of AKT3 by miR-122 over-expression decreased Bad phosphorylation, increased total Bad accumulation, elevated cleaved caspase 3 levels, and induced programmed cell death. This miR-122 induced apoptosis was rescued by partially restoring AKT3 expression, indicating that AKT3 is not only essential in regulating cellular migration, but also plays pivotal roles in apoptosis and proliferation. Therefore, restoration of miR-122 can induce anti-tumor activities through specific targeting of AKT3, suggesting that miR-122 can function as a tumor suppressor in HCCs which harbor diminished miR-122 expression.

The tumor suppressor functions of miR-122 restoration were observed in all three HBV transformed cell lines tested (Hep3B2, SNU-182, and SNU-475). Interestingly, in the hepatoblastoma cells tested (HepG2), AKT3 is not expressed even though miR-122 is highly down regulated. Interestingly, this cell line is not as aggressive or tumorigenic as the HCC transformed cell lines. This suggests that this cell lines likely lacks the mechanism necessary for tumorigenesis and down regulation of miR-122 is not sufficient to induce that change. Even though miR-122 and AKT3 expression are inversely correlated in the HBV-transformed cell lines tested, whether this correlation is specifically related to the HBV-transformation needs to be investigated in more detail.

In conclusion, we have shown that miR-122 directly and specifically binds to the 3’UTR of human AKT3, and over-expression of miR-122 in HBV-transformed HCC cell lines is able to decrease AKT3, at both the transcript and protein level, to block cell migration, induce apoptosis, and inhibit cell proliferation and tumor growth in mice. Ectopically expressed AKT3 is able to rescue these anti-tumor characteristics induced by miR-122 over-expression indicating that the regulation of tumorigenesis by miR-122 is mediated through targeting AKT3 in these HCCs.

## Materials and Methods

### Cell Culture

All cell lines (except for Huh-7 which was acquired from Japan’s Health Science Research Resource Bank) were procured from the American Type Culture Collection (ATCC) and maintained in Dulbecco’s modified Eagle’s medium (DMEM) containing 10% fetal bovine serum (FBS) supplemented with L-glutamine and grown in a humidified incubator with 5% CO_2_ at 37°C.

### Stable cell line generation

We used the System Biosystem’s LentimiR™ vectors, which consist of the native stem loop structure, for stable expression of our miRNAs. The lentiviral expression vector contains the genetic elements responsible for packaging, transduction, stable integration of the viral expression construct into genomic DNA, and expression of the specific mature miRNAs. For production of a high titer of viral particles, we used the ViraPower™ Lentiviral Support Kits (Invitrogen) together with Lipofectamine™ 2000 (Invitrogen) for tranfecting the vectors into HEK293T cells. Because infected cells stably express copGFP, we used FACS sorting to select for the infected cells harboring the miRNA of interest.

### RT-PCR

TaqMan miRNA assays (Life Technologies, CA) were used to quantify the expression levels of mature miR-122 as well mRNAs for AKT1, 2, 3. Total RNA extracted by miRvana (life technologies) was reverse transcribed in reaction mixture containing miR-specific stem-loop RT primers. Quantitative real time polymerase chain reaction (qPCR) was performed in triplicate reactions containing the prepared cDNA and TaqMan specific primers in Universal Master Mix without AmpErase UNG (Applied Biosystems). The qPCR was conducted at 95°C for 10 minutes, followed by 40 cycles of 95°C for 15 seconds and 60°C for 60 seconds in a 7900 Real Time PCR machine (Applied Biosystem) and threshold cycles (*C*_T_) were calculated using Sequence Detection Software (SDS v2.2.1, Applied Biosystem). All mRNA quantification data were normalized to 18S RNA. All miRNA data are expressed relative to a RNU48 small nuclear (sn) RNA TaqMan PCR performed on the same samples, unless otherwise specified. Fold expression was calculated from the mean *C*_T_ values using the 2^−ΔΔCt^ method.

### Immunoblotting

Cells were lysed in buffer containing 50 mM NaCl, 1.5 mM MgCl_2_, 50 mM HEPES, 10% glycerol, 1 mM EGTA, 1% Triton X-100, 0.5% NP-40 supplemented with 1 mM Na_3_VO_4_, 1 mM PMSF, 1 mM NaF, 1 mM β-glycerophosphate. Protease inhibitor cocktail (Roche) and phosphatase inhibitor cocktail (Roche) was added prior to use. Protein concentration was determined using the BCA Protein Assay (Pierce/Thermo Fisher Scientific) following the manufacturer’s instructions. Protein (30–50 µg) was resolved by SDS-PAGE and transferred onto nitrocellulose membrane. Blots were probed with primary antibodies to detect proteins of interest. After incubation with secondary antibodies, membranes were visualized by chemiluminescence (Pierce/Thermo Fisher Scientific). All antibodies were from Cell Signaling Technology, Inc with the exception of Actin and AKT2 (Santa Cruz Biotechnology).

### Cell proliferation, apoptosis, and migration assays

Resazurin Fluorescent Assay was used for the proliferation assays. Briefly, Cells are seeded at 3000–5,000 cells/100 ul/well in DMEM +10% FBS in a 96 well plate, and were incubated overnight at 37°C in 5% CO_2_. Resazurin (Sigma) fluorescent dye was added (1∶100) to each well. The cells were incubated at 37°C in 5% CO2 for 4 hours at which point the plate was read for fluorescence at 530/590 nm on the HTS 7000 plate reader. Cell Signaling Technologies PathScan® Apoptosis Multi-Target Sandwich ELISA Kits were used in the apoptosis assays. Briefly, antibodies for cleaved caspase 3 and phosphorylated BAD had been coated onto microwells by the manufacturer. After incubation with the cell lysates, the target protein was captured by the coated antibodies. Following extensive washing, a detection antibody was added to detect the captured target protein. An HRP-linked secondary antibody was then used to recognize the bound detection antibody. HRP substrate, TMB, was finally added for color development which is proportional to the quantity of bound target protein. Cell Biolab’s CytoSelect™ Cell Migration Assay Kit containing polycarbonate membrane inserts (8 µm pore size) in a 24-well plate was used in our migration assays. Migratory cells are able to extend protrusions towards HGF (Hepatic Growth Factor), and pass through the pores of the polycarbonate membrane. Non-migratory cells are removed from the top of the membrane and the migratory cells are stained and quantified.

### Transfection of DNA constructs and miR-122 mimics

The entire 3′UTR of the hsa-AKT3 gene was amplified from a human cDNA clone obtained from Origene using the following primers incorporating the *Nhe*I and *Sal*I restriction sites: AKT3 3′UTR forward, CGGCTAGCCGCGTCTCTTTCATTCTGCTACTTCACTGTC; AKT3 3′UTR reverse, CCGGTCGACCGCTTCACTCAGGTAGAAATATGAAAAAGAAGG **.** The AKT3 3′UTR amplicon was ligated into the pmirGLO Dual-Luciferase miRNA target expression vector (Promega) between the *Nhe*I and *Sal*I restriction sites. Transfection of DNA constructs into cell lines was performed using Lipofectamin 2000 reagent (Life Technologies) according to the manufacturer's protocols. The double-stranded RNA that mimics endogenous human miR-122a, and a scrambled miRNA used as a non-targeting control, were obtained from Dharmacon. The introduction of miRNA mimics was accomplished by lipofection using Lipofectamine (Life Technologies), with a 30 nM miRNA mimic concentration per condition.

### Luciferase assay

Three days after transfection with appropriate constructs, the cells were lysed and processed for luciferase luminescence measurements. For detection of luciferase activity the Dual-Glo luciferase assay system (Promega) was used as described by the manufacturer. Briefly, an appropriate amount of Dual-Glo reagent was added to the cell medium enabling cell lysis and subsequent detection of firefly luminescence in a luminometer. Normalization of the samples were performed by addition of the Dual-Glo Stop & Glo reagent enabling the detection of renilla luminescence (measured to normalize data for transfection efficiency variability), and the luciferase activity in relative light units (RLU) was subsequently calculated.

### Statistics

Quantitative data are presented as the mean ± SD. Student's *t* test was used to determine significant differences between two groups. One-way ANOVA with Bonferroni's multiple comparison test was used to analyze significant differences among multiple groups; *p*≤0.05 was considered significant unless otherwise stated.

### Animal studies

Six to eight-week-old nu/nu athymic female mice were obtained from Jackson Labs; the mice were maintained in pressurized ventilated caging at the Pfizer La Jolla animal facility. All studies were done under the approval of Pfizer Institutional Animal Care and Use Committee’s guidelines. Tumors were established by injecting 5×10^6^ cells suspended 1:1 (v/v) with reconstituted basement membrane (Matrigel, BD Biosciences). Tumor dimensions were measured with vernier calipers, and tumor volumes were calculated using this formula: π/6 x (larger diameter) x (smaller diameter)^2^. Tumor growth inhibition percentage (TGI %) was calculated as 100 x (1-▵T/▵C). One way ANOVA Statistical analysis were performed and noted as *** for p value is less than 0.001.
